# Diagnostic value of serum HE4 in endometrial cancer: a meta-analysis

**DOI:** 10.1186/1477-7819-12-169

**Published:** 2014-05-29

**Authors:** Yachun Bie, Zhenyu Zhang

**Affiliations:** 1 Department of Obstetrics and Gynecology, Beijng Chao-yang Hospital affiliated to Capital Medical University, 100020 Beijing, P. R. China

**Keywords:** Endometrial cancer (EC), Serum, HE4, Diagnoses, Meta-analysis

## Abstract

**Background:**

Endometrial cancer (EC) is a common female malignant cancer. The age of incidence has become younger than before. If the diagnosis is during stage I, then the survival rate is about 90%. To date, there are no specific tumor markers for endometrial cancer. We usually use serum CA125 to help in diagnosing it. However, a serum biomarker CA125 greater than 35 U/ml is not useful in diagnosing EC at an early stage. Now, human epididymis protein 4 (HE4) has been intensively studied, and has been described as a new marker for ovarian cancer. The goal of this study was to evaluate the clinical value of serum HE4 in the diagnosis of endometrial cancer by meta-analysis.

**Methods:**

We used MEDLINE, EMBASE, Cochrane Library and CBM databases to search the literature. The meta-analysis was performed by using Meta-Disc 1.4 software.

**Results:**

All data we obtained showed that the major advantage of HE4 lies in its specificity in endometrial cancer diagnosis. Its sensitivity in serum was not as high as expected. But this evidence is not enough.

**Conclusions:**

Additional studies, particularly to evaluate HE4’s capability in identifying EC at an early stage, will be needed.

## Background

Endometrial cancer is a common female malignancy. The incidence varies because of different lifestyles and regions. In developed countries, the incidence rate is the highest among female genital malignancies, and the age of incidence has become younger than before. The prognosis is closely related to the disease stage. If the diagnosis is during stage I, then the survival rate is about 90%.

There are no specific tumor markers for endometrial cancer. CA125 was detected in 1983 by Bast *et al*. [1] as the epithelial ovarian carcinoma antigen. It is a macromolecular polymer glycoprotein, expressed in body cavity epithelial. Serum CA125 level is elevated in many primary tumors, such as ovarian, endometrial, colorectal, breast and lung cancers. It is also elevated in a number of other conditions, including pregnancy, inflammation, endometriosis, fibroids, benign ovarian cysts, cirrhosis and abdominal surgery [2]. It can be detected in the blood, pleural effusion, ascites and amniotic fluid. So, as a tumor marker, it has low sensitivity and specificity for early diagnosis of endometrial carcinoma. Several authors have found that higher serum CA125 levels correlated with the extra uterine disease and advanced cases. It is always used as a marker to evaluate prognosis and recurrence in endometrial cancer. However,a CA125 level greater than 35 U/ml is not useful in diagnosing early stages of endometrial cancer (EC).

It may be necessary to find other biomarkers for early detection of endometrial cancer and for monitoring high risk patients, such as those with severe obesity, diabetes, Lynch syndrome (hereditary non-polyposis colorectal cancer syndrome), *PTEN* gene defects or those given tamoxifen therapy for breast cancer. New biomarkers will also be used to guide treatment, monitor therapeutic effect and predict recurrence. To date, human epididymis protein 4 (HE4) has been intensively studied. It was identified in the epithelium of the distal epididymis and originally predicted to be a protease inhibitor involved in sperm maturation [3]. Now it has been described as a new marker for ovarian cancer [4]. RG Moore *et al*. has proved serum HE4 is elevated in all stages of endometrial cancer and is more sensitive in early stage endometrial cancer compared to CA125 [5].

The goal of this study was to evaluate the clinical value of serum HE4 in the diagnosis of endometrial cancer by meta-analysis.

## Methods

Literature searches of MEDLINE, EMBASE, the Cochrane Library databases and CBM were performed. Index words included the medical subject headings (MeSH): endometrial neoplasms and uterine neoplasms, and the following text words: endometrium, endometrial, uterus, uterine, cancer, carcinoma, HE4, WFDC2, human epididymis protein 4 and human epididymis-specific protein 4. Search terms related to study design and publication type included systematic review, clinical trial, meta-analysis, controlled clinical trials and randomized controlled trials. Reference lists of identified studies were scanned for additional citations until no additional articles could be identified.

Inclusion criteria were all papers with pathological diagnosis and serum HE4 value. And the aim of these articles was the role of serum HE4 in diagnosis of endometrial cancer.

Reviews and papers without a serum HE4 test value were excluded. Studies reporting insufficient data for the construction of a two-by-two table were excluded from the final analyses.

### Quality assessment

The methodological quality of each trial was evaluated by the quality-assessment tool for diagnostic accuracy studies (QUADAS-2). The quality of research was evaluated independently by two reviewers, based on the following criteria: 1) the experiment has a pathological diagnosis, 2) the inclusion criteria of the research were clear, 3) statistics were appropriate, 4) the study can be repeated, 5) the study shows a correct threshold, and 6) biases in the study were discussed.

### Statistical analyses

The meta-analysis was performed by using Meta-Disc 1.4 software (The program has been developed by the Unit of Clinical Biostatistics team of the Ramón y Cajal Hospital in Madrid (Spain)). Analysis of heterogeneity between studies was done using the χ^2^ test. If there was no significant heterogeneity between studies (*P* > 0.1, *I*^2^ ≤ 50%), the analysis was performed using a fixed-effects model and analyzed bias to obtain sensitivity, specificity, positive predictive and negative predictive values. If there was statistical heterogeneity among studies, the analysis was performed using the random-effects model (*P* ≤ 0.1, *I*^2^ > 50%).

## Results

The search identified 34 potentially relevant papers based on the search terms. A total of six studies met all the eligibility criteria for this review. The selection process for articles included in the meta-analysis is shown in Figure 1. Basic information on included studies is shown in Table 1.

**Figure 1:** Selection process for articles included in the meta-analysis.

**Table 1:** Summary data of the original studies

**Author**	**Country**	**Year**	**Type of study**	**Patients**	**Control**	**Cut off (pmol/L)**	**TP**	**FP**	**FN**	**TN**	**SEN**	**SPE**
Moore RG *et al*. [5]	USA	2008	prospective/retrospective	171	156	/	78	8	93	148	46	95
Zanotti L *et al*. [6]	Italy	2012	retrospective	193(152 + 41)	125	51	152	19	41	106	79	85
						64	127	6	66	119	66	95
Angioli R *et al*. [7]	Italy	2013	prospective	101(95 + 6)	103	70	60	0	41	103	59	100
						150	36	0	65	103	36	100
Omer B*et al*. [8]	Turkey	2013	prospective l	64(54 + 10)	94(60 + 34)	60	48	32	16	62	75	66
Bignotti E *et al*. [9]	Italy	2011	prospective	138(109 + 29)	76	/	92	4	46	72	67	95
Zhang, Ai-min *et al*. [10]	China	2012	prospective	124	206(97 + 109)	/	51	10	73	196	41	95
**Total**				791	760							

Studies [6], [7], [8] and [9] included patients with different pathological types. The pathological types of patients in study [5] and study [10] are unclear. Studies [8] and [10] included people with uterine benign disease and had healthy people as controls. The controls of other studies are healthy.

FN, False Negative; FP, False Positive; SEN, Sensitivity; SPE, Specificity TN, True Negative; TP, True Positive.

In the six trials there are one retrospective study [6], four prospective studies and one study analyzed as having either prospective or retrospective data [5].

In control groups, Angioli *et al*. [7] was the first to enroll patients with benign uterine disease as controls. Omer *et al*. [8] used patients with benign uterine disease and healthy women as controls. Moore *et al*. [5] and Bignotti *et al*. [9] used postmenopausal healthy women as controls in their studies. And also an article in Chinese used patients with benign uterine disease and healthy women as controls [10]. Moreover, three studies evaluated the sensitivity of HE4 without indicating a cut-off value [5,9,10]. And two other studies reported data on two thresholds [6,7]. We have included the two-by-two tables for all reported thresholds.

Four articles clearly showed pathological types in the patient groups [6-9].

### Meta-analysis

High levels of heterogeneity lay in both sensitivity (I^2^ = 92.9%) and specificity (I^2^ = 93.1%). Forest plots of sensitivity and specificity of HE4 for EC prediction were shown in Figures 2 and 3. Mean estimates and their 95% CIs were: sensitivity 0.594 (0.564 to 0.623), specificity 0.920 (0.901 to 0.936). A threshold effect existed (Spearman correlation coefficient: 0.755, *P*-value = 0.031). The random-effects model was used to pool estimates. And heterogeneity existed among the study designs. Cochran-Q is 22.13 in a diagnostic odds ratio, *P* = 0.0024 (Figure 4). The area under the summary receiver operating-characteristic curve (SROC) was 0.8321 (Figure 5). The DOR (diagnostic odds ratio) is 20.816 (11.434 to 37.896).

**Figure 2:** **Forest plots of sensitivity of HE4 for EC prediction.** The red circles represent the sensitivity of one study; the black line shows its confidence interval. If a study reported accuracy data for more than one cut-off, its results are included more than once.

**Figure 3:** **Forest plots of specificity of HE4 for EC prediction.** The red circles represent the specificity of one study; the black line shows its confidence interval. If a study reported accuracy data for more than one cut-off, its results were included more than once.

**Figure 4:** **Diagnostic odds ratio of HE4 for EC prediction.** Heterogeneity existed among the study designs. Cochran-Q is 22.13 in diagnostic odds ratio, *P* = 0.0024. Heterogeneity existed among the studies’ designs. Cochran-Q is 22.13 in diagnostic odds ratio, *P* = 0.0024.

**Figure 5:** **SROC of HE4 for EC prediction.** Each circle represents each study in the meta-analyses. The size of each study is indicated by the size of the circle. The regression summary receiver operating characteristic curves summarize the overall diagnostic accuracy.

Meta-regression was used to investigate the potential sources of heterogeneity. We found the control group (healthy women or women with benign disease) and the different pathological types of patients act as potential sources of heterogeneity. We divided the studies into different subgroups according to pathological types of patients and whether they included people with uterine benign diseases as controls. Then subgroup analysis was made and heterogeneity was assessed in these subgroups (Table 2).

**Table 2:** Effect of subgroups

**Subgroup**		**Studies**	**SEN (95% CI)**	**SPE (95% CI)**	**DOR (95% CI)**	**I**^**2**^**(%)**	***P***
**Pathological types of patients**	Adenocarcinoma + other types	6	0.652 (0.618 to 0.685)	0.903 (0.877 to 0.925)	27.291 (11.011 to 67.640)	77.10	0.001
	Unclear	2	0.437 (0.380 to 0.496)	0.950 (0.923 to 0.970)	14.524 (8.547 to 24.681)	0.00	0.817
**Control**	Uterine benign diseases + healthy	4	0.500 (0.449 to 0.551)	0.917 (0.889 to 0.940)	22.555 (5.473 to 92.943)	80.10	0.002
	Healthy	4	0.646 (0.609 to 0.682)	0.923 (0.896 to 0.945)	23.426 (15.767 to 34.806)	3.50	0.375
**Total**		8	0.594 (0.564 to 0.623)	0.920 (0.901 to 0.936)	20.816 (11.434 to 37.896)	68.40	0.0024

The studies were divided into different subgroups according to the patients’ pathological types and different controls. DOR, Diagnostic odds ratio; SEN, Sensitivity; SPE, Specificity.

## Discussion

Several reviews have been published in recent years about using serum HE4 for the diagnosis of EC. Most of these reviews, however, are based on non-systematic methods [11-14].

The result of our meta-analysis show that serum HE4 level could help predict the presence of EC based on whether the area under the curve (AUC) was 0.8321. HE4 showed sensitivity 0.594(0.564 to 0.623) and high specificity 0.920(0.901 to 0.936). Therefore, the associated poor sensitivity of HE4 clearly limits its value in its diagnosis of EC. This conclusion is similar to that of Jacob *et al*. [15], in which the authors concluded the major advantage of HE4 lies in its specificity and improved detection of borderline tumors and early stage ovarian and tubal cancers. They also showed that there were no benefits from combining HE4 and CA125 as ovarian tumor markers in a clinical setting [15].

However, due to the heterogeneity, the meta-analysis results should be interpreted with caution. We used meta-regression and found the control group (healthy women or women with benign disease) and the different pathological types of patients act as potential sources of heterogeneity. We also noted that the overall diagnostic accuracy of HE4 is more superior in healthy control groups compared to control subjects with benign disease (Table 2). The limitation of the present meta-analysis is that there is no unified cutoff. The assay method (ELISA, chemiluminescent micro particle immunoassay, bead-based array system), and the patients’ status and small samples also account for the lack of evidence to support HE4 as a tumor marker for EC. Some studies found that HE4 levels in healthy subjects are associated with age and smoking status. Age-dependent reference limits are suggested [14,16]. It is necessary to collect more data to improve the research. And it would be essential to define a specific normal range and cut-off value for women of different ages, respectively.

## Conclusion

This review showed that although we do have an estimate of the test accuracy of serum HE4 for the diagnosis of EC, we have not enough data to estimate its value in clinical practice. It is necessary to get more data to improve the quality of the research. Additional studies, particularly to evaluate HE4 role in endometrial cancer staging and pathological types, are needed.

## Abbreviations

CI: Confidence interval; DOR: Diagnostic odds ratio; EC: Endometrial cancer; HE4: Human epididymis protein 4; SROC: summary receiver operating-characteristic curve.

## Competing interests

No conflict of interest exits in the submission of this manuscript, and manuscript is approved by all authors for publication.

## Authors’ contributions

All authors have contributed significantly and all authors are in agreement concerning the content of the manuscript. YB and ZZ evaluated the researches independently. YB drafted the manuscript. All authors read and approved the final manuscript.
